The article "Hsa_circ_0000673 is down-regulated in gastric cancer and inhibits the proliferation and invasion of tumor cells by targetting miR-532-5p" was retracted in 2022. Reasons: duplicated images; original data or images not available.

# Hsa_circ_0000673 is down-regulated in gastric cancer and inhibits the proliferation and invasion of tumor cells by targetting miR-532-5p

**DOI:** 10.1042/BSR20180538

**Published:** 2018-09-19

**Authors:** Peng Chang, Furong Wang, Yumin Li

**Affiliations:** 1 School of Life Sciences, Lanzhou University, Lanzhou 730000, China; 2 Lanzhou University Second Hospital, Lanzhou 730000, China; 3 Department of General Surgery, Lanzhou University Second Hospital, Lanzhou 730000, China; 4 Department of Pathology, Lanzhou University Second Hospital, Lanzhou 730000, China; 5 The Key Laboratory of the Digestive System Tumors of Gansu Province, Lanzhou University Second Hospital, Lanzhou 730000, China

**Keywords:** cell proliferation, gastric cancer, Hsa_circ_0000673, Invasion, miR-532-5p

## Abstract

Circular RNAs (circRNAs), a new class of endogenous non-coding RNAs, have recently been known to play critical roles in various cellular biological processes, including tumorigenesis, in which they act as an miRNA sponge that regulates gene expression. Thus, revealing the functions of circRNAs in carcinogenesis and cancer development has been of great interest. However, their expression and functions in gastric cancer (GC) development are still largely unknown. Therefore, the present study aimed to identify novel deregulated circRNAs in GC and reveal their biological functions and molecular mechanisms in GC. Quantitative real-time PCR (qRT-PCR) was performed to measure the expression levels of circRNAs in GC tissues, cell lines, and plasma. The MTT assay, colony formation assay, transwell assay, and tumor xenografts *in vivo* were used to evaluate the effects of circRNAs on the proliferation and invasion of GC. The abovementioned methods coupled with Western blotting were used to investigate the molecular mechanisms. The current study showed that hsa_circ_0000673 was significantly down-regulated in GC. Overexpression of hsa_circ_0000673 inhibited the proliferation and invasion of GC cells. In contrast, hsa_circ_0000673 down-regulation promoted the proliferation and invasion of GC cells. Further studies revealed that hsa_circ_0000673 targetted miR-532-5p and up-regulated the expression of RUNX3. The present study showed that hsa_circ_0000673 was decreased in GC and it exerted tumor-suppressing effects by targetting miR-532-5p and up-regulating RUNX3 expression level. Hsa_circ_0000673 may be a promising diagnosis biomarker and therapeutic target in GC.

## Introduction

Gastric cancer (GC) is a common malignant tumor with the fourth highest occurrence amongst all cancers and is the second leading cause of cancer-related deaths worldwide [1,2]. Many Asian countries have high incidence of GC, especially China and Japan [3,4]. From 2009 to 2011, 679100 patients were diagnosed with GC in China, of which 498000 died [4]. Despite advanced diagnostic techniques and therapeutic strategies, the prognosis of GC remains poor [5]. The occurrence and development of GC are complex biological processes accompanied by the activation of oncogenes or dysregulation of tumor suppressor genes [6–10]. Thus far, the molecular mechanism underlying gastric carcinogenesis has not been fully understood. Further elucidation on the molecular mechanism underlying GC development is beneficial in identifying new diagnostic and therapeutic targets.

Circular RNAs (circRNAs), closed-loop RNAs produced through end-to-end joining of RNA transcription fragments during transcription, are a new class of endogenous non-coding RNAs [11,12]. Although circular transcripts have been known for at least 40 years, they were once considered as aberrant RNA splicing or specific pathogens [13]. However, studies suggested that circRNAs participate in a variety of physiological and pathological processes, including acting as miRNAs sponge in the development of cancer [14,15]. In addition, unlike other non-coding RNAs, circRNAs are very stable due to their ring structure [16]. A research has shown that circRNAs are found in the plasma, platelets, and exosomes, and therefore are useful as potential biomarkers for cancer diagnosis and therapy [17]. Further elucidation on the deregulated circRNAs in cancers and identification of their functions will help improve the diagnosis and treatment of cancers.

In the present study, we analyzed circRNAs expression level in GC tissues and plasma to confirm hsa_circ_0000673 circRNA down-regulation in GC cell lines, and also examined its correlation with GC staging. We also performed further studies to confirm whether hsa_circ_0000673 can target miR-532-5p and up-regulate RUNX3, thus suppressing GC proliferation and invasion. In the current study, we proposed hsa_circ_0000673 as a biomarker for diagnosis and as a potential therapeutic target for GC treatment.

## Materials and methods

### Tissue and blood specimens

All patients with GC in the present study were histopathologically and clinically diagnosed at the Lanzhou University Second Hospital (Lanzhou, China) from 2015 to 2017. Patients’ age ranged from 25 to 60 years. The ratio of male to female patients was 1:1. All patients were of Han ethnicity from Gansu Province. No patient received pre-operative chemotherapy, radiotherapy, or target therapy. All tumor tissues were histologically confirmed as GC using Hematoxylin and Eosin (H&E) staining after surgical resection. The clinicopathologic staging of the patients were in accordance with the manual by the American Joint Committee on Cancer. Normal gastric tissues 3 cm from the margin of resected neoplastic tissues of patients with GC were isolated and confirmed by pathological evaluation. We also collected 38 plasma samples from 14 healthy donors and 24 patients with GC. Consistent with the inclusion criteria of patients with GC, healthy donors were aged 25–60 years and of Han ethnicity from Gansu Province, with a male to female ratio of 1:1. They had no history of stomach or other systematic diseases and they were recruited from the hospital at the same time as patients with GC. We obtained approval from the Institutional Research Ethics Committee and written informed consent from all participants for use of tissue and blood specimens in our study.

### Microarray data analysis

Two human circRNA microarray data (GSE83521 and GSE78092) were downloaded from NCBI GEO DataSets. circRNAs with more than two-folds change in expression level in tumor and normal counterparts were chosen for further investigation. We used CircBase (http://www.circbase.org/) to unify all circRNAs’ names. Then, we used Venny 2.1 (http://bioinfogp.cnb.csic.es/tools/venny/index.html) to filter out circRNAs with the same trend in GSE83521 and GSE78092. The sequence of circRNAs can be obtained in CircBase.

### Cell lines and cell culture

The GC cell lines AGS, MKN28, BGC823, MKN45, HGC-27, MGC803, and SGC7901, as well as the normal gastric epithelial cell line and HEK-293 T cells were purchased from the Cell Bank of Type Culture Collection (Shanghai City, China). These cell lines were cultured in RPMI-1640 medium (Invitrogen, Carlsbad, CA) supplemented with 10% FBS (Gibco, Carlsbad, CA, U.S.A.) and 1% penicillin/streptomycin (Invitrogen). The cells were incubated at 37°C and 5% CO_2_.

### RNA extraction and RT-qPCR

Total RNA was isolated from the tissue specimens and cultured cells using an RNeasy Plus Mini Kit (Qiagen, Chatsworth, CA). Plasma RNA was isolated with a miRNeasy Serum/Plasma Kit (Qiagen, Chatsworth, CA) according to the manufacturer’s instructions. cDNA was synthesized by reverse transcription using an MMLV transcriptase (Promega) using random primers. For gene detection, real-time RT-PCR was performed on a LC480 real-time PCR detection system (Bio-Rad) using a Roche SYBR FAST Universal qPCR Kit (Roche Molecular Biochemicals). GAPDH was used as an internal control. The sequences of primers are presented in Table 1.

**Table 1:** The list of primers and siRNA sequences

Gene	Forward primer	Reverse primer
**qRT-PCR primer**		
hsa_circ_0000673	GTATAGGTGGAACAGTCTTAA	TTATATTCCTTCTTTAGAGTTTGG
RSL1D1	AAGGCAGTGGACGCTCTCT	AGGAGTTGAATTGGGTTCATCC
hsa_circ_0074854	ATGAACAGATGACTAAGT	ATCCACATTAAGTTGAGA
hsa_circ_0009172	GGACTATCTTCCTTCGTT	GCTACCACTTTCTTCTGA
GAPDH	GGAGCGAGATCCCTCCAAAAT	GGCTGTTGTCATACTTCTCATGG
**Clone primer**		
pLCDH-ciR-0000673	ATCTGTTCAATTAACGAATTCtgaaatatgctatcttacAGATTATCTCCCTCCAAACTC	TCATCCCAAATTAGTGGATCCtcaagaaaaaatatattcACCTGCAAGAACCACTTTTAG
**siRNA for hsa_circ_0000673**	**siRNA sequence**	
001	AAAGTGGTTCTTGCAGATTATdTdT	
002	AGTGGTTCTTGCAGATTATCTdTdT	
003	TTGCAGATTATCTCCCTCCAAdTdT	

Abbreviation: qRT-PCR, quantitative real-time PCR.

### Plasmids and transfection

The complete sequence of hsa_circ_0000673 was obtained from circBase. We purchased the retroviral transfer plasmid pLCDH-ciR-puro from Geneseed (Guangzhou, China). Then, we designed circRNA primers based on the pLCDH-ciR-puro manual. The PCR product was inserted into pLCDH-ciR-puro with ClonExpress® II purchased from Vazyme (Jiangsu, China). Sequencing and identification were needed to design two primers in the middle of the target circRNA fragment, bidirectional cross-sequencing, and the interval between the two primers should not be shorter than 90 bp. siRNAs of hsa_circ_0000673 were synthesized by RiboBio (Guangzhou, China), designed to target the junction region of hsa_circ_0000673 sequence. miR-532-5p mimics, anti-miR-532-5p oligonucleotides, and their corresponding control oligonucleotides were also purchased from RiboBio (Guangzhou, China). Transfection of plasmids or oligonucleotides was performed using Lipofectamine® 3000 reagent (Invitrogen, Carlsbad, CA) according to the manufacturer’s instructions. The sequences of clone primers and siRNA are presented in Table 1.

### Luciferase report assay

HEK-293 T cells (8 × 10^4^) were seeded in 48-well plates and cultured for 24 h. Then, miR-532-5p mimics, LUC-hsa_circ_0000673 and LUC-hsa_circ_0000673-mutant reporter plasmid and pRL-TK plasmid (Promega) were co-transfected in HEK-293 T cells using Lipofectamine® 3000 reagent (Invitrogen, Carlsbad, CA) according to the manufacturer’s instructions. After 48 h, we detected the luciferase activities of these reporters in whole cell lysate and normalized to corresponding luciferase activities of pRL-TK through the Dual-Luciferase Reporter Assay System (Promega) according to the manufacturer’s protocols.

### Western blot analysis

Western blot analysis was performed according to a previously described standard method [18] using anti-RUNX3 (1:500; Abcam, Cambridge, MA), anti-P21 (1:500; Cell Signaling, Danvers, MA), anti-BIM (1:500; Cell Signaling) or anti-GAPDH antibodies (1:3000; Cell Signaling).

### Cell proliferation assays

Cell proliferation ability was assessed using the MTT assay and clone formation assay. For MTT assay, the cells were seeded in 96-well plates (800 cells/well). Cell proliferation was detected every 24 h according to the manufacturer’s protocol. Briefly, 20 µl MTT solution (Sangon Biotech, China) was added to each well, which was incubated at 37°C for 4 h. Next, the supernatant was discarded and 150 µl DMSO was added to each well. The mixture was then gently shaken at room temperature for 15 min. The solution was measured spectrophotometrically at 450 nm. For clone formation assay, the cells were seeded in six-well plates (400 cells/well) and cultured for 10 days at 37°C and 5% CO_2_. The supernatant was discarded and the cells were gently washed with 1 ml 1× PBS. Next, the supernatant was discarded again and 1 ml paraformaldehyde was added to each well. The mixture was gently shaken at room temperature for 15 min. The paraformaldehyde was discarded afterward and 1 ml 0.1% Crystal Violet was added to each well. The mixture was then gently shaken at room temperature for 15 min. The Crystal Violet was discarded and the cells were washed with ddH_2_O and air-dried in a ventilated place. The number of clones formed was counted by ImagePro Plus 6.0 software. Each experiment was repeated at least three times.

### Transwell assays

Cell invasion ability was assessed using the transwell assay. The transwell assay was performed according to a previously described standard method [19].

### Tumor xenografts *in vivo*

The cells (2 × 10^6^ cells) were subcutaneously implanted in the inguinal folds of 7-week-old BALB/c nude mice (*n*=3 per group). Tumor lengths (L) and widths (W) were measured every 5–7 days. Tumor volumes were calculated using the following equation: volume (mm^3^) = L*W^2^/2. At the experimental end point, mice were anesthetized and killed. Tumors were then removed and photographed.

### Statistical analysis

Statistical analysis was conducted using the Student’s *t*test. All error bars represent the mean ± S.D. of three independent experiments. All statistical analyses were performed using the GraphPad Prism 5.0 software package (GraphPad Software, Inc., San Diego, U.S.A.). *P-*values <0.05 were considered statistically significant.

## Results

### Hsa_circ_0000673 expression is significantly down-regulated in GC

To identify novel circRNAs involved in the development of GC, we integrated two human circRNA microarray data (GSE83521 and GSE78092, downloaded from GEO DataSets) to screen common differentially expressed genes. We found that hsa_circ_0000673, hsa_circ_0009172, and hsa_circ_0074854 were all significantly down-regulated in GC tissues, compared with those in non-tumor tissues (Figure 1A). Further, we determined the expression levels of hsa_circ_0000673, hsa_circ_0009172, and hsa_circ_0074854 in several GC cell lines and human GC tissues by using quantitative real-time PCR (qRT-PCR). As shown in Figure 1B,C and Supplementary Figure S1A,B, the expression levels of hsa_circ_0000673 and hsa_circ_0074854 were significantly down-regulated in the GC cell lines and GC tissue samples than in the normal human gastric epithelial cell line GES-1 and the normal gastric epithelial cells samples, respectively. However, both *in vitro* and *in vivo*, there was no significant difference in the expression level of hsa_circ_0009172 between GC and normal cells (Supplementary Figure S1C,D). We selected hsa_circ_0000673 for further investigations, whereas hsa_circ_0074854 was studied by other researchers in our facility.

**Figure 1:** Hsa_circ_0000673 is down-regulated in GC tissue, cell lines, and plasma (**A**) Screening of common differentially expressed circRNAs in two human GC circRNA microarray data (GSE83521 and GSE78092). (**B**) Analysis of hsa_circ_0000673 expression in normal human gastric epithelial cells (GES-1 cell line) and cultured GC cell lines by qRT-PCR. (**C**) Analyses of hsa_circ_0000673 expression levels in 36 pairs of primary GC tissues (T) and their corresponding adjacent non-cancerous tissues (N). (**D**) Analysis of hsa_circ_0000673 expression in GC tissues of various clinical stages. (**E**) Comparison of plasma hsa_circ_0000673 levels in healthy donors and patients with GC. Error bars represent the mean ± S.D. of three independent experiments. The statistical analysis was performed using the two-tailed Student’s *t* test (*P<0.05).

To determine the clinical significance of hsa_circ_0000673 expression level in patients with GC, we measured the expression level of hsa_circ_0000673 in 64 human GC specimens by using qRT-PCR. The specimens comprised 25 cases of stage I, 23 cases of stage II, and 16 cases of stages III and IV. As shown in Figure 1D, the expression level of hsa_circ_0000673 was significantly decreased with the increase in GC stage. As previous studies have shown that circRNA stably exists in the plasma, we further determined hsa_circ_0000673 expression in 38 plasma samples collected from 14 healthy donors and 24 patients with GC. As shown in Figure 1E, plasma hsa_circ_0000673 was significantly down-regulated in patients with GC, compared with that in healthy donors (*P*<0.001). Taken together, the above data suggested that hsa_circ_0000673 expression was significantly down-regulated in GC.

### Overexpression of hsa_circ_0000673 inhibited the proliferation and invasion of GC cells *in vitro*

To address the role of hsa_circ_0000673 in GC pathogenesis, we established the GC cell lines AGS and BGC823, which exhibited low endogenous hsa_circ_0000673 expression levels, as cell lines that stably overexpress hsa_circ_0000673. As shown in Supplementary Figure S2A, the expression levels of hsa_circ_0000673 were markedly increased in hsa_circ_0000673-overexpressing GC cells compared with the corresponding vector control cells. On the genome, hsa_circ_0000673 is located in chr16:11940357-11940700, which is also a part of the gene *RSL1D1*. We subsequently measured the mRNA level of RSL1D1 by using qRT-PCR to evaluate the effect of hsa_circ_0000673 overexpression on RSL1D1. As shown in Supplementary Figure S2A, hsa_circ_0000673 overexpression did not affect *RSL1D1* mRNA level.

Furthermore, using the abovementioned established cell lines, we examined the effect of hsa_circ_0000673 on GC cell proliferation and invasion. As shown in Figure 2A, the proliferation curves determined by MTT assays showed that the overexpression of hsa_circ_0000673 significantly attenuated growth in cancer cells compared with that in the normal cells. In addition, using colony formation assay (Figure 2B), we revealed that AGS-circ-0000673 and BGC823-circ-0000673 formed fewer and smaller colonies than the vector group. Moreover, as shown in Figure 2C, the invasive ability of GC cells was remarkably decreased by hsa_circ_0000673 overexpression. Taken together, these data showed that hsa_circ_0000673 overexpression significantly inhibited the proliferation and invasion of GC cells.

**Figure 2:** Overexpression of hsa_circ_0000673 suppresses GC cell proliferation and invasion (**A**) MTT assay revealed cell growth curves of AGS and BGC823 cell lines. (**B**) Representative micrographs (left) and relative quantitation (right) of Crystal Violet-stained cell colonies analyzed by colony formation assay for 10 days. (**C**) Representative images (left) and relative quantitation (right) of invading cells in response to hsa_circ_0000673 overexpression using Transwell assays. Error bars represent mean ± S.D. derived from three biologically independent experiments. A two-tailed Student’s *t* test was used for statistical analysis (*P<0.05).

### Down-regulation of hsa_circ_0000673 promoted the proliferation and invasion of GC cells *in vitro*

We performed hsa_circ_0000673 silencing by RNAi-mediated knockdown in MGC803 cells, which exhibited relatively high endogenous hsa_circ_0000673 expression, to evaluate whether endogenous hsa_circ_0000673 inhibit the proliferation and invasion of GC cells. As shown in Supplementary Figure S2B, hsa_circ_0000673 expression was significantly down-regulated by siRNAs compared with that of the negative control group. However, hsa_circ_0000673 silencing did not affect the expression level of RSL1D1 (Supplementary Figure S2B).

As shown in Figure 3A,B, endogenous hsa_circ_0000673 silencing markedly enhanced the proliferation and clone formation capacity of GC cells. Moreover, as shown in Figure 3C, endogenous hsa_circ_0000673 silencing also enhanced the invasive ability of GC cells. Taken together, these data further showed that hsa_circ_0000673 inhibited the proliferation and invasion of GC cells.

**Figure 3:** Silencing endogenous hsa_circ_0000673 promotes GC cell proliferation and invasion (**A**,**B**) MTT and colony formation assays were performed to measure the proliferation ability of MGC803 cells transfected with si-hsa_circ_0000673 compared with si-NC. (**C**) Representative images (left) and relative quantitation (right) of invading cells in response to hsa_circ_0000673 silencing with Transwell assays. Error bars represent mean ± S.D. derived from three biologically independent experiments. A two-tailed Student’s *t*test was used for statistical analysis (*P<0.05). Abbreviation: NC, negative control.

### Hsa_circ_0000673 inhibits the tumor growth of GC cells *in vivo*

To examine the effect of hsa_circ_0000673 on GC growth *in vivo*, we established a line of stable hsa_circ_0000673-silenced GC cells, namely MGC803-circ-0000673 sh3 cells. (Supplementary Figure S2C). Next, we subcutaneously implanted AGS-vector, AGS-circ-0000673, MGC803-scramble, or MGC803-circ-0000673 sh3 cells into the inguinal fold of athymic mice. As shown in Figure 4A, the hsa_circ_0000673-overexpressing cells developed tumors at a significantly slower rate than that of the vector control cells within the second week following inoculation, and the difference in average tumor volume between the experimental and control animals continued to decrease by 2.1-fold at the experimental end point (day 35). In parallel, a decrease in tumor size was also observed (Figure 4B). In contrast, hsa_circ_0000673-silenced cells developed larger tumor at a faster rate than scramble control cells (Figure 4C,D). Taken together, these data suggested that hsa_circ_0000673 strongly inhibited the tumor growth of GC cells *in vivo*.

**Figure 4:** Hsa_circ_0000673 suppresses the tumor growth of GC cells *in vivo* (**A**,**B**) A total of 2 × 10^6^ AGS-vector and AGS-circ-0000673 were implanted in BALB/c nude mice (*n*=3 per group). (A) Tumor growth curves in mice inoculated with AGS cells at indicated days. (B) At the experimental end point, tumors were dissected and photographed as indicated. (**C**,**D**) A total of 2 × 10^6^ MGC803-scramble and MGC803-circ-0000673 sh3 were implanted in BALB/c nude mice (*n*=3 per group). Tumor growth curves were shown in (C) and the tumors’ photo taken at the experimental end point was shown in (D). Data were presented as mean ± S.D. (*n*=3 mice/group). Student’s *t*test was used for statistical analysis (*P<0.05).

### Hsa_circ_0000673 targetted miR-532-5p and up-regulated RUNX3

Evidence has shown that circRNAs sequester miRNAs to terminate the regulation of their target genes. To investigate the mechanism underlying the effect of hsa_circ_0000673 on the inhibition of proliferation and invasion in GC cells, we searched for miRNAs associated with hsa_circ_0000673. By combining the prediction from the databases TargetScan and MiRanda, we selected miR-532-5p as a potential target of hsa_circ_0000673 (Figure 5A). To figure out whether hsa_circ_0000673 can bind with miR-532-5p, we synthesized an hsa_circ_0000673 fragment which contained the predicted binding site and another hsa_circ_0000673 fragment which predicted that binding site was mutant. Then, we inserted them immediately downstream of the luciferase reporter gene separately (p-LUC-hsa_circ_0000673 and p-LUC-hsa_circ_0000673-mutant). If miR-532-5p can bind with hsa_circ_0000673, transfection of miR-532-5p can inhibit the luciferase activity. As shown in Figure 5B, in contrast with negative control (NC), transfection of miR-532-5p can significantly decrease the luciferase activity when the corresponding target sites were wild-type. However, transfection of miR-532-5p has no significant effect on luciferase activity when the corresponding target sites were mutated from the luciferase reporter. To further determine the relationship between hsa_circ_0000673 and miR-532-5p, we measured the expression level of miR-532-5p in hsa_circ_0000673-overexpressed or -silenced GC cells by using qRT-PCR. As shown in Figure 5C,D, hsa_circ_0000673 significantly decreased the expression of miR-532-5p. In addition, we detected the expression of miR-532-5p in the GC cell lines and GC tissues by using qRT-PCR. As shown in Figure 5E,F, miR-532-5p was significantly up-regulated in the GC cell lines and GC tissue samples compared with that in the GES-1 cell line and the normal tissue samples, respectively. And miR-532-5p expression level was significantly increased with the increase in GC stage (Figure 5G). These results (Figure 5E–G) were consistent with previous studies. Combined with the results shown in Figure 1, we found that GC exhibited opposite trends in the expression levels of hsa_circ_0000673 and miR-532-5p. Previous research shows that miR-532-5p functions as an oncogenic miRNA that promotes cell growth, migration, and invasion in human GC cells by directly down-regulating the expression levels of RUNX3 and its targets. To further verify the effect of hsa_circ_0000673 on miR-532-5p, we examined the expression levels of RUNX3 and its downstream effectors (p21, Bim, E-cadherin). Through Western blotting analysis (Figure 5H), we showed that hsa_circ_0000673 significantly increased the protein levels of RUNX3, p21, Bim, and E-cadherin in AGS and BGC823 cells, whereas the opposite occurred in the hsa_circ_0000673-knockdown MGC803 cells. These results confirmed that miR-532-5p as an hsa_circ_0000673-associated miRNA in GC cells. Hsa_circ_0000673 targetted miR-532-5p and up-regulated the expression of RUNX3 and its downstream effectors.

**Figure 5:** Hsa_circ_0000673 up-regulates RUNX3 by targetting miR-532-5p (**A**) Predicted binding site of hsa_circ_0000673 and miR-532-5p. (**B**) Luciferase reporter assay for the luciferase activity of LUC-hsa_circ_0000673 or LUC-hsa_circ_0000673-mutant in HEK-293 T cells co-transfected with miR-532-5p mimics. (**C**) The results of qRT-PCR showed that hsa_circ_0000673 overexpression significantly decreased the miR-532-5p level. (**D**) Silencing hsa_circ_0000673 significantly up-regulated the expression of miR-532-5p. (**E**) Analysis of miR-532-5p expression in normal human gastric epithelial cells (GES-1 cell line) and cultured GC cell lines by qRT-PCR. (**F**) Analyses of miR-532-5p expression levels in 36 pairs of primary GC tissues (T) and their corresponding adjacent non-cancerous tissues (N). (**G**) Analysis of miR-532-5p expression in GC tissues with different clinical stages. (**H**) The impact of hsa_circ_0000673 on miR-532-5p downstream targets were analyzed by Western blotting. Error bars represent mean ± S.D. derived from three biologically independent experiments. A two-tailed Student’s *t* test was used for statistical analysis (*P<0.05).

### Hsa_circ_0000673 inhibited the proliferation and invasion of GC cells by regulating miR-532-5p

To ascertain the role of miR-532-5p in the hsa_circ_0000673-induced inhibition of GC cell proliferation and invasion, we transiently transfected miR-532-5p mimics into the hsa_circ_0000673-overexpressed AGS and BGC823 cells, and miR-532-5p inhibitors into the hsa_circ_0000673-silenced MGC803 cells. As shown in Figure 6A,B, miR-532-5p transduction significantly reversed the hsa_circ_0000673-induced inhibition of cancer cell growth in AGS and BGC823 cells, whereas miR-532-5p-silencing by miR-532-5p inhibitors significantly decreased the hsa_circ_0000673-induced inhibition of cancer growth rate of in MGC803 cells. Through the transwell assay, (Figure 6C,D) we also showed that miR-532-5p significantly reversed the hsa_circ_0000673-induced inhibition of GC cells invasion. Furthermore, through Western blotting assay (Figure 6E), we showed that miR-532-5p significantly reversed the hsa_circ_0000673-mediated up-regulation of RUNX3 and its downstream effectors. Taken together, these data strongly suggested that hsa_circ_0000673 inhibited the proliferation and invasion of GC cells by regulating miR-532-5p.

**Figure 6:** miR-532-5p is required for hsa_circ_0000673-induced inhibition of proliferation and invasion in GC (**A**,**B**) The results of MTT assays determined that miR-532-5p can significantly reverse the growth inhibition of hsa_circ_0000673 in GC cells. (**C**,**D**) The results of Transwell assays showed that miR-532-5p can significantly reverse hsa_circ_0000673-induced inhibition of invasion in GC cells. (**E**) Western blotting assays showed that miR-532-5p significantly reverse hsa_circ_0000673-mediated up-regulation of RUNX3 and its downstream effectors. Error bars represent mean ± S.D. derived from three biologically independent experiments. A two-tailed Student’s *t* test was used for statistical analysis (*P<0.05).

## Discussion

Recently, the function of circRNAs in carcinogenesis and cancer development has garnered much attention. However, their expression level and function in GC development are still largely unknown, with only a few circRNAs reported to be involved in the development of GC [20–29]. In our present study, we analyzed two human circRNA microarray data, GSE83521 and GSE78092, and identified a novel circRNA significantly down-regulated in GC, namely hsa_circ_0000673. Further experimental studies suggested that hsa_circ_0000673 overexpression inhibited the proliferation and invasion of GC cells. In contrast, hsa_circ_0000673 silencing significantly promoted the proliferation and invasion of GC cells. To date, the expression and function of hsa_circ_0000673 in tumor development and progression remains unclear. We revealed for the first time that hsa_circ_0000673 was significantly decreased in GC and it exerted tumor-suppressing effects.

Despite suggesting tumor-suppressing effects of hsa_circ_0000673 in GC, the present study did not investigate other important deregulated circRNAs involved in the development of GC due to the screening we conducted at the beginning of the study. At the same time, interestingly, we found that almost all circRNAs reported in GC are decreased. Hence, in future studies, we will focus on identifying other highly expressed circRNAs in GC or determining the mechanism underlying the down-regulation of most circRNAs in GC.

A recent study has shown that circRNAs exert their functions through multiple ways, including miRNA sponge, RBP sponge, and mRNA regulator [30]. In our present study, we found that hsa_circ_0000673 potentially functioned as a sponge of oncogenic miR-532-5p that up-regulated RUNX3, p21, and Bim expression levels, as well as consequently suppressed the proliferation and invasion of GC. A previous study has shown that miR-532-5p is overexpressed in GC [31]. However, the mechanism of the high expression of miR-532-5p in GC is still unclear. Our current study showed that the down-regulation of hsa_circ_0000673 may play an important role in the high expression of miR-532-5p in GC.

Compared with other non-coding RNAs, such as miRNAs and long non-coding RNAs (lncRNAs), circRNAs are highly conserved and stable. These two important properties of circRNAs were possibly responsible for their potential as ideal biomarkers in the diagnosis and therapy of cancers. In the present study, we collected 38 plasma samples, including 14 from healthy people and 24 from patients with GC, and detected the plasma level of hsa_circ_0000673 in these samples. The result showed that plasma hsa_circ_0000673 level was significantly down-regulated in patients with GC (*P*<0.001), suggesting that hsa_circ_0000673 may be useful as diagnosis biomarkers and therapeutic target in GC.

In summary, hsa_circ_0000673 expression was significantly decreased in GC and negatively correlated with GC stage. Functionally and mechanistically, hsa_circ_0000673 inhibited GC proliferation and invasion through the sponge effect on miR-532-5p and up-regulation of RUNX3 expression, indicating its role as a tumor suppressor in GC development. Furthermore, plasma hsa_circ_0000673 level was significantly down-regulated in patients with GC, suggesting the potential roles of hsa_circ_0000673 as a diagnosis biomarker and therapeutic target in GC.

## Supporting information

**Supplemental Fig. 1:** A. Analysis of hsa_circ_0074854 expression in normal human gastric epithelial cells (GES-1) and cultured GC cell lines by qRT-PCR. B. Analyses of hsa_circ_0074854 expression levels in 36 pairs of primary GC tissues (T) and their corresponding adjacent noncancerous tissues (N) by qRT-PCR. C. Analysis of hsa_circ_0009172 expression in normal human gastric epithelial cells(GSE-1) and cultured GC cell lines by qRT-PCR. D. Analyses of hsa_ hsa_circ_0009172 expression levels in 36 pairs of primary GC tissues (T) and their corresponding adjacent noncancerous tissues (N) by qRT-PCR.

**Supplemental Fig. 2:** A. Stable overexpression of hsa_circ_0000673 in AGS and BGC823 cell lines was confirmed by qRT-PCR. Overexpression of hsa_circ_0000673 didn’t affect the expression level of RSL1D1, the linear RNA isomer of hsa_circ_0000673. B. The results of qRT-PCR determined that the relative expression of hsa_circ_0000673 decreased by transfection with si-hsa_circ_0000673 in MGC803 cells, compared with the transfection with si-NC. Silencing hsa_circ_0000673 didn’t affect the expression level of RSL1D1. C. The results of qRT-PCR showed that we successfully established hsa_circ_0000673 stable-silenced GC cells. Silencing hsa_circ_0000673 didn’t affect the expression level of RSL1D1. Error bars represent mean ± SD derived from three biologically independent experiments. A two-tailed Student’s t-test was used for statistical analysis (* P<0.05). NC, negative control.

## Abbreviations

circRNA: circular RNA
GC: gastric cancer
qRT-PCR: quantitative real-time PCR

## References

[1] TorreL.A., BrayF., SiegelR.L., FerlayJ., Lortet-TieulentJ. and JemalA. (2015) Global cancer statistics, 2012. CA Cancer J. Clin. 65, 87–108 10.3322/caac.21262 25651787

[2] FerlayJ., SoerjomataramI., DikshitR., EserS., MathersC., RebeloM. (2015) Cancer incidence and mortality worldwide: sources, methods and major patterns in GLOBOCAN 2012. Int. J. Cancer 136, E359–386 10.1002/ijc.29210 25220842

[3] CharvatH., SasazukiS., InoueM., IwasakiM., SawadaN., ShimazuT. (2016) Prediction of the 10-year probability of gastric cancer occurrence in the Japanese population: the JPHC study cohort II. Int. J. Cancer 138, 320–331 10.1002/ijc.29705 26219435

[4] FuS.J., ZhaoQ., JiF., ChenM.G., WuL.W., RenQ.Q. (2016) Elevated preoperative serum gamma-glutamyltranspeptidase predicts poor prognosis for hepatocellular carcinoma after liver transplantation. Sci. Rep. 6, 28835 10.1038/srep28835 27381639PMC4933871

[5] DuraesC., AlmeidaG.M., SerucaR., OliveiraC. and CarneiroF. (2014) Biomarkers for gastric cancer: prognostic, predictive or targets of therapy? Virchows Arch. 464, 367–378 10.1007/s00428-013-1533-y 24487788

[6] QiX., ZhangD.H., WuN., XiaoJ.H., WangX. and MaW. (2015) ceRNA in cancer: possible functions and clinical implications. J. Med. Genet. 52, 710–718 10.1136/jmedgenet-2015-103334 26358722

[7] HuangK.K., RamnarayananK., ZhuF., SrivastavaS., XuC., TanA.L.K. (2018) Genomic and epigenomic profiling of high-risk intestinal metaplasia reveals molecular determinants of progression to gastric cancer. Cancer Cell 33, 137–150.e135, 10.1016/j.ccell.2017.11.01829290541

[8] HayakawaY., AriyamaH., StancikovaJ., SakitaniK., AsfahaS., RenzB.W. (2015) Mist1 expressing gastric stem cells maintain the normal and neoplastic gastric epithelium and are supported by a perivascular stem cell niche. Cancer Cell 28, 800–814 10.1016/j.ccell.2015.10.003 26585400PMC4684751

[9] PadmanabhanN., UshijimaT. and TanP. (2017) How to stomach an epigenetic insult: the gastric cancer epigenome. Nat. Rev. Gastroenterol. Hepatol. 14, 467–478 2851363210.1038/nrgastro.2017.53

[10] SongS.H., JeonM.S., NamJ.W., KangJ.K., LeeY.J., KangJ.Y. (2018) Aberrant GATA2 epigenetic dysregulation induces a GATA2/GATA6 switch in human gastric cancer. Oncogene 37, 993–1004 10.1038/onc.2017.397 29106391

[11] MemczakS., JensM., ElefsiniotiA., TortiF., KruegerJ., RybakA. (2013) Circular RNAs are a large class of animal RNAs with regulatory potency. Nature 495, 333–338 10.1038/nature11928 23446348

[12] ChenL.L. and YangL. (2015) Regulation of circRNA biogenesis. RNA Biol. 12, 381–388 10.1080/15476286.2015.1020271 25746834PMC4615371

[13] SangerH.L., KlotzG., RiesnerD., GrossH.J. and KleinschmidtA.K. (1976) Viroids are single-stranded covalently closed circular RNA molecules existing as highly base-paired rod-like structures. Proc. Natl. Acad. Sci. U.S.A. 73, 3852–3856 10.1073/pnas.73.11.38521069269PMC431239

[14] HuangH., WangX.P., LiX.H., ChenH., ZhengX., LinJ.H. (2017) Prognostic value of pretreatment serum alanine aminotransferase/aspartate aminotransferase (ALT/AST) ratio and gamma glutamyltransferase (GGT) in patients with esophageal squamous cell carcinoma, BMC Cancer. 17, 544, 10.1186/s12885-017-3523-y28806937PMC5556356

[15] WangX., ZhangY., HuangL., ZhangJ., PanF., LiB. (2015) Decreased expression of hsa_circ_001988 in colorectal cancer and its clinical significances. Int. J. Clin. Exp. Pathol. 8, 16020–16025 26884878PMC4730091

[16] JeckW.R., SorrentinoJ.A., WangK., SlevinM.K., BurdC.E., LiuJ. (2013) Circular RNAs are abundant, conserved, and associated with ALU repeats. RNA 19, 141–157 10.1261/rna.035667.112 23249747PMC3543092

[17] LiY., ZhengQ., BaoC., LiS., GuoW., ZhaoJ. (2015) Circular RNA is enriched and stable in exosomes: a promising biomarker for cancer diagnosis. Cell Res. 25, 981–984 10.1038/cr.2015.82 26138677PMC4528056

[18] WangY., JiaL. and WuC.Y. (2008) Triptolide inhibits the differentiation of Th17 cells and suppresses collagen-induced arthritis. Scand. J. Immunol. 68, 383–390 10.1111/j.1365-3083.2008.02147.x 18782267

[19] CaiJ., ZhaoJ., ZhangN., XuX., LiR., YiY. (2015) MicroRNA-542-3p suppresses tumor cell invasion via targeting AKT pathway in human astrocytoma. J. Biol. Chem. 290, 24678–24688 10.1074/jbc.M115.649004 26286747PMC4598981

[20] TianM., ChenR., LiT. and XiaoB. (2018) Reduced expression of circRNA hsa_circ_0003159 in gastric cancer and its clinical significance. J. Clin. Lab. Anal. 32, 10.1002/jcla.22281PMC681715428618205

[21] ChenS., LiT., ZhaoQ., XiaoB. and GuoJ. (2017) Using circular RNA hsa_circ_0000190 as a new biomarker in the diagnosis of gastric cancer. Clin. Chim. Acta 466, 167–171 10.1016/j.cca.2017.01.025 28130019

[22] XieY., ShaoY., SunW., YeG., ZhangX., XiaoB. (2018) Downregulated expression of hsa_circ_0074362 in gastric cancer and its potential diagnostic values. Biomark. Med. 12, 11–20 10.2217/bmm-2017-0114 29240459

[23] ShaoY., ChenL., LuR., ZhangX., XiaoB., YeG. (2017) Decreased expression of hsa_circ_0001895 in human gastric cancer and its clinical significances. Tumour Biol. 39, 10.1177/101042831769912528443463

[24] SunH., TangW., RongD., JinH., FuK., ZhangW. (2018) Hsa_circ_0000520, a potential new circular RNA biomarker, is involved in gastric carcinoma. Cancer Biomark 21, 299–306 10.3233/CBM-170379 29103021PMC13078270

[25] ZhangC., WangH., NingZ., XuL., ZhuangL., WangP. (2017) Serum liver enzymes serve as prognostic factors in patients with intrahepatic cholangiocarcinoma. Onco. Targets Ther. 10, 1441–1449 10.2147/OTT.S12416128331337PMC5348058

[26] ChenJ., LiY., ZhengQ., BaoC., HeJ., ChenB. (2017) Circular RNA profile identifies circPVT1 as a proliferative factor and prognostic marker in gastric cancer. Cancer Lett. 388, 208–219 10.1016/j.canlet.2016.12.006 27986464

[27] ZhangJ., LiuH., HouL., WangG., ZhangR., HuangY. (2017) Circular RNA_LARP4 inhibits cell proliferation and invasion of gastric cancer by sponging miR-424-5p and regulating LATS1 expression. Mol. Cancer 16, 151 10.1186/s12943-017-0719-3 28893265PMC5594516

[28] HuangM., HeY.R., LiangL.C., HuangQ. and ZhuZ.Q. (2017) Circular RNA hsa_circ_0000745 may serve as a diagnostic marker for gastric cancer. World J. Gastroenterol. 23, 6330–6338 10.3748/wjg.v23.i34.6330 28974900PMC5603500

[29] LaiZ., YangY., YanY., LiT., LiY., WangZ. (2017) Analysis of co-expression networks for circular RNAs and mRNAs reveals that circular RNAs hsa_circ_0047905, hsa_circ_0138960 and has-circRNA7690-15 are candidate oncogenes in gastric cancer. Cell Cycle 16, 2301–2311 10.1080/15384101.2017.1380135 28980874PMC5788484

[30] LasdaE. and ParkerR. (2014) Circular RNAs: diversity of form and function. RNA 20, 1829–1842 10.1261/rna.047126.114 25404635PMC4238349

[31] XuX., ZhangY., LiuZ., ZhangX. and JiaJ. (2016) miRNA-532-5p functions as an oncogenic microRNA in human gastric cancer by directly targeting RUNX3. J. Cell. Mol. Med. 20, 95–103 10.1111/jcmm.12706 26515139PMC4717862

